# ANPrAod: Identify Antioxidant Proteins by Fusing Amino Acid Clustering Strategy and *N*-Peptide Combination

**DOI:** 10.1155/2021/5518209

**Published:** 2021-04-08

**Authors:** Qilemuge Xi, Hao Wang, Liuxi Yi, Jian Zhou, Yuchao Liang, Xiaoqing Zhao, Yongchun Zuo

**Affiliations:** ^1^State Key Laboratory of Reproductive Regulation and Breeding of Grassland Livestock, College of Life Sciences, Inner Mongolia University, Hohhot 010070, China; ^2^Agronomy College, Inner Mongolia Agricultural University, Hohhot, Inner Mongolia 010019, China; ^3^Biotechnology Research Centre, Inner Mongolia Academy of Agricultural and Animal Husbandry Science, Hohhot 010021, China

## Abstract

Antioxidant proteins perform significant functions in disease control and delaying aging which can prevent free radicals from damaging organisms. Accurate identification of antioxidant proteins has important implications for the development of new drugs and the treatment of related diseases, as they play a critical role in the control or prevention of cancer and aging-related conditions. Since experimental identification techniques are time-consuming and expensive, many computational methods have been proposed to identify antioxidant proteins. Although the accuracy of these methods is acceptable, there are still some challenges. In this study, we developed a computational model called ANPrAod to identify antioxidant proteins based on a support vector machine. In order to eliminate potential redundant features and improve prediction accuracy, 673 amino acid reduction alphabets were calculated by us to find the optimal feature representation scheme. The final model could produce an overall accuracy of 87.53% with the ROC of 0.7266 in five-fold cross-validation, which was better than the existing methods. The results of the independent dataset also demonstrated the excellent robustness and reliability of ANPrAod, which could be a promising tool for antioxidant protein identification and contribute to hypothesis-driven experimental design.

## 1. Introduction

High concentrations of reactive oxygen species will result in oxidative damage to proteins, DNA/RNA, and the polyunsaturated fatty acids, which in turn can lead to hypertension, cancer, coronary heart disease, and Alzheimer's disease [1–4]. Antioxidant proteins eliminate excess free radicals through interactions to protect cells and DNA from oxidative damage, which is closely related to disease control, so they have become a research hotspot in the field of life science and pharmacology [5, 6]. The method of identifying antioxidant proteins through biochemical experiments has problems of being time-consuming and expensive, so there is an urgent need to develop related computation methods to complement the experiments.

In recent years, with the mass production of protein sequences, a series of methods have been developed to identify different types of proteins. Based on a support vector machine (SVM), Zuo et al. successfully predicted defensin proteins with an accuracy of 92.38% [7, 8]. Feng et al. designed a predictor called Aodpred to identify antioxidant proteins, with a cross-validation accuracy of 74.79% [9]. Fu et al. proposed a method called StackCPPred, which used a stack-based machine learning method to effectively predict cell-penetrating peptides [10]. Tan et al. applied the binomial distribution method to recode the sequence to predict hormone-binding protein [11]. Research on these machine learning methods yielded promising results, but there were some limitations in predicting the accuracy and efficiency of antioxidant proteins.

In this study, a novel feature extraction method, the amino acid reduction alphabets combined with the *N*-peptide composition strategy was used to identify antioxidant proteins. Amino acid-reduced alphabets are often used for large-scale protein structure analysis and prediction [8, 12, 13]. It can tolerate many changes in sequences while still retaining the basic folding and function of the proteins.  Figure 1 shows the ANPrAod framework flow. First, a strict benchmark dataset was constructed to ensure the validity of the comparison among models. Subsequently, amino acid reduction alphabets combined with *N*-peptide composition (*N* = 1, 2, 3) strategy was used to extract the feature vectors and compare them to obtain the optimal scheme. Based on the support vector machine (SVM), ANPrAod yielded an accuracy of 87.53% in the fivefold cross-validation which was better than the existing methods through a series of comparison results. Finally, the prediction performance of ANPrAod was objectively evaluated on the independent dataset and principal component analysis (PCA), which proved the robustness and reliability of the model. In conclusion, ANPrAod was an effective tool for predicting antioxidant proteins, which could assist experimental studies of treatment-related diseases.

## 2. Materials and Methods

### 2.1. Dataset

The premise of building a high-quality model is to use a reliable database [14–16]. To facilitate the comparison of our model with previous work, we used the same benchmark dataset collected in the study of Feng et al. [9, 17]. Finally, 1805 protein sequences were used as the training dataset, including 253 antioxidant proteins and 1552 nonantioxidant proteins. In addition, a strictly independent dataset was constructed by us, containing 240 protein sequences (50 antioxidant proteins and 190 nonantioxidant proteins) from Uniprot to objectively evaluate the robustness of the model.

### 2.2. Support Vector Machine

The support vector machine includes four main kernel functions: linear kernel function, polynomial kernel function, radial basis function (RBF), and sigmoid kernel function [18]. The core of SVM is to transform the data into high-dimensional Hilbert space and find the optimal separation hyperplane. For the convenience of scientific research, Chang and Lin developed the LIBSVM package, which can be downloaded for free from the following location http://www.csie.ntu.edu.tw/~cjlin/libsvm/ [19]. It has been used in computational biology [20–22].

In this study, the LIBSVM package with RBF kernel was used to predict antioxidant proteins. We used the grid search to optimize the regularization parameter *C* and the kernel parameter *γ* to improve the performance of the model. The selection ranges of *C* and *γ* are as follows:

(1) $$\begin{array}{c} 2^{-5}<C<2^{15},\\ 2^{-15}<\gamma <2^{3}. \end{array}$$

### 2.3. Reduced Amino Acid Alphabets

Researchers have shown that the amino acid sequence can be redefined according to the position, structure, function, and similarity of the amino acid in the protein sequences which are called reduced amino acid alphabets [23]. Compared to original protein sequences, the reduced amino acid alphabets performed superior predictive ability in reducing protein complexity and extracting conservative features hidden in noise signals [24]. Based on RAACBook, we adopted 673 amino acid reduction schemes to be applied to our model [25, 26].

### 2.4. *N*-Peptide Composition

Single amino acid interactions and more detailed sequence information can be effectively mined by *N*-peptide (*N* = 1, 2, 3) composition. We did not try longer *N*-peptide because of our memory limitation [8, 27]. For a natural protein sequence, the dipeptide composition can be described as follows:

(2) $$\begin{array}{c} P=R_{1}R_{2}R_{3}\cdots R_{L-1}R_{L},\\ F={\left[d_{1},d_{2},\cdots ,d_{400}\right]}^{T}, \end{array}$$

where *R*_1_ represents the first amino acid in the protein sequence, *L* represents the total length of the protein sequence. *d*_*i*_ (*i* = 1, 2, ⋯, 400) is the *i*th dipeptide in the 400 amino acid combination, and *T* means the transposition operator.

### 2.5. Feature Selection

Feature selection is an important step in building a powerful model, which is of great significance for improving the performance of the classifier [28–30]. Analysis of variance (ANOVA), which measures the variance of features by calculating the ratio of features between and within groups, helps us evaluate the weight of each feature and is widely used in bioinformatics [31, 32]. Appropriate dimensional features could save computing resources, reduce the risk of overfitting, and improve prediction accuracy, so we used incremental feature selection (IFS) to filter features measured by analysis of variance to train the model [33]. The ANOVA formula is defined as follows:

(3) $$\begin{array}{c} F=\frac{S_{x}^{2}}{S_{\gamma }^{2}},\\ S_{X}^{2}=\frac{1}{n-1}\overset{n}{\underset{i=1}{\sum }}{\left(x_{i}-\overset{¯}{x}\right)}^{2},\\ S_{y}^{2}=\frac{1}{m-1}\overset{m}{\underset{i=1}{\sum }}{\left(y_{i}-\overset{¯}{y}\right)}^{2}, \end{array}$$

where *F* is the variance value of the feature, *S*_*X*_^2^ is the sample variance between groups, and *S*_*y*_^2^ denotes the sample variance within groups.

### 2.6. Performance Evaluation

The traditional metrics, sensitivity (Sn), specificity (Sp), accuracy (Acc), and area under the receiver operating characteristic curve (AUC), were used to evaluate the performance of the models, which are defined as follows [20–22, 34–37]:

(4) $$\begin{array}{c} \text{Sn}=\frac{\text{TP}}{\text{TP}+\text{FN}},\\ \text{Sp}=\frac{\text{TN}}{\text{TN}+\text{FP}},\\ \text{Acc}=\frac{\text{TP}+\text{TN}}{\text{TP}+\text{FN}+\text{TN}+\text{FP}},\\ \text{AUC}=\underset{i}{\sum }\left\{\left(1-\beta_{i}\right)\cdot \Delta \alpha +\frac{1}{2}\left[\Delta \left(1-\beta \right)\cdot \Delta \alpha \right]\right\}, \end{array}$$

where

(5) $$\begin{array}{c} \Delta \left(1-\beta \right)=\left(1-\beta_{i}\right)-\left(1-\beta_{i-1}\right),\\ \Delta \alpha =a_{i}-a_{i-1}, \end{array}$$

where TP, TN, FP, and FN represent true positive, true negative, false positive, and false negative of samples, respectively. *α*_*i*_ and *β*_*i*_ (*i* ∈ *N*) are the false positive rate and false negative rate obtained by different thresholds. The receiver operating curve (ROC) was used by us to quantitatively evaluate the performance of the model [38]. The true positive rate and false positive rate are the *x*-axis and *y*-axis, respectively.

## 3. Results

### 3.1. Performance of Different Reduced Amino Acid Alphabets

RAACBook summarizes the 673 amino acid reduced alphabets and classifies them into 74 types; each type contains 2-19 reduced sizes [25]. Based on SVM, the protein sequences of the training dataset were reduced according to RAACBook, and the *N*-peptide (*N* = 1, 2, 3) composition was used to extract feature vectors to evaluate the influence of different feature extraction methods on the predictive performance of the model. Figures 2(a) and 2(b) show the accuracy density profiles of 673 reduced amino acid cluster models for predicting antioxidant proteins with different *N*-peptide compositions (*K* = 1, 2, 3). Excitedly that compared with the combination of single peptide and tripeptide, dipeptide has achieved better accuracy performance, which meant that they can significantly simplify complexity and reduce information redundancy. Therefore, we further analyzed all the detailed accuracy of the dipeptide combination and showed 22 types with the optimal calculation results using the heatmap. It can be seen from Figures 3(a) and 3(b) that in type 19 and size 10, the accuracy of fivefold cross-validation reached 87.31%, which has the optimal discriminative ability.

### 3.2. Determination of Optimal Features

It is well known that the predictive power of the model does not improve linearly with the increase of feature dimensions, so it is necessary to examine the predictive performance of different feature sets in dipeptide combinations (type 19, size 10). First, we used ANOVA to score each feature by weight, then sorted them according to the score from largest to smallest. Then, the IFS (step size is 1) was used to determine the optimal number of features. From Figure 3(c), when the top 93 features were used, the model accuracy has the highest fivefold cross-validation result of 87.53%. Finally, the optimal feature set was used by us to construct the SVM model for antioxidant protein prediction. The ROC curve drawn according to the fivefold cross-validation result of the optimal feature set was used to further objectively evaluate the performance of ANPrAod (Figure 4(a)).

### 3.3. Feature Analysis

The information maximization method of information theory was used by Solis to polymerize amino acids into 2-19 groups (Table 1) [39]. Mutual information was maximized based on the similarity of the paired contact interactions of the 20 amino acids, and then, this was used as the objective function to mimic the natural paired contact that occurs in natural proteins [39]. Specifically, they are assigned according to nonpolar aromatic (FWY), nonpolar aliphatic and sulfur-containing (CILMV), acid (DE), basic (HR), small (AT), and other polarities (NQS), which also demonstrate that these alphabets maintain the ability to identify remote interactions.

### 3.4. Comparison with Previous Methods

To demonstrate the superiority of ANPrAod in the identification of antioxidant proteins, we compared it with published methods. As shown in Table 2, based on the same dataset, the fivefold cross-validation results showed that ANPrAod has the optimal performance with an accuracy of 87.53%, which was better than other methods. This is due to the motivation that SVM was originally designed for binary classification and the theoretical bounds from generalization error [40]. The upper bound of generalization error does not depend on the dimension of space, and the maximum boundary is used to minimize the error boundary to minimize the distance between the hyperplane of two classes and the nearest data point [41]. In addition, ANPrAod used only 93 features compared to 158 features used by AodPred, which reduced computational complexity and the risk of overfitting. This comparison demonstrated the effectiveness of the amino acid reduction alphabets combined with *N*-peptide combination strategy and the strong function of ANPrAod to identify antioxidant proteins.

### 3.5. Performance Assessment of ANPrAod on Independent Dataset

It is not rigorous to evaluate the model only based on the information in the training set, which may overestimate the performance of the model. In order to avoid this problem, we tested ANPrAod on an independent dataset to evaluate its real performance. The confusion matrix results showed that ANPrAod still achieved excellent prediction results, which proved the robustness and effectiveness of the model and could be a powerful tool to assist the study of antioxidant proteins (Figure 4(b)). In addition, we compared the natural protein sequences with the reduced amino acid protein sequences by using PCA, which further confirmed the superiority of the amino acid reduction combined with the *N*-peptide composition strategy (Figures 4(c) and 4(d)).

## 4. Conclusion

Feature extraction is extremely important for generalization ability; it can promote the subsequent learning of the model and has better interpretability [10, 42]. In this study, a new feature representation scheme of amino acid reduction alphabets combined with *N*-peptide combination strategy was applied to redefine protein sequences. The new feature vectors were used to train SVM to find the optimal scheme for predicting antioxidant proteins. The accuracy of fivefold cross-validation was 87.53%, and the ROC curve area was 0.7266, which was better than other models. PCA and independent dataset results also indicated that the amino acid reduction alphabets combined with *N*-peptide combination strategy can effectively reduce the data complexity, and ANPrAod has strong robustness to accurately predict antioxidant proteins. We anticipated that ANPrAod can accurately and rapidly identify antioxidant proteins based on peptide sequence and promote the development of related drug research. In future work, we will establish an online web server and extend the research content to other fields.

## Figures and Tables

**Figure 1:** The workflow of ANPrAod predictor.

**Figure 2:** Binary accuracy density maps. (a) Based on amino acid reduced alphabets, binary precision density map of different *N*-peptide combinations (*N* = 1, 2, 3). (b) Based on amino acid reduced alphabets, Acc univariate density map of different *N*-peptide combinations (*N* = 1, 2, 3).

**Figure 3:** Evaluation of predictive performance of antioxidant proteins. (a) Fivefold cross-validation results of different feature representation schemes. (b) The prediction accuracy of the optimal size in different types. (c) The IFS curve showed that under the dipeptide combination (type = 19, size = 10), the accuracy was up to 87.53% when using the top 93 features.

**Figure 4:** The ROC curve of ANPrAod and its performance on independent dataset. (a) ROC curve of ANPrAod constructed by the optimal feature set. (b) ANPrAod prediction confusion matrix in independent dataset. (c) PCA for natural independent dataset. (d) PCA of independent datasets processed by amino acid reduction alphabets.

**Table 1:** Amino acid alphabet reduction using the information maximization device.

Size	Cluster
2	CFILMVWY-ADEGHKNPQRST
3	CFILMVWY-DEGKNQS-AHPRT
4	FWY-CILMV-DEGKNQS-AHPRT
5	FWY-CILMV-DEGKNS-APQT-HR
6	FWY-CILMV-DE-GKNQS-APT-HR
7	FWY-CILMV-DE-K-GNPQS-AT-HR
8	FWY-ILMV-C-DE-K-GNPQS-AT-HR
9	FWY-ILMV-C-DE-K-GNQS-PT-A-HR
10	WY-F-ILMV-C-DE-K-GNQS-PT-A-HR
11	WY-F-ILMV-C-DE-K-G-PNQS-T-A-HR
12	WY-F-IL-MV-C-DE-K-G-PNQS-T-A-HR
13	WY-F-IL-MV-C-DE-K-G-P-NQS-T-A-HR
14	W-Y-F-IL-MV-C-DE-K-G-P-NQS-T-A-HR
15	W-Y-F-IL-MV-C-DE-K-G-P-NQS-T-A-H-R
16	W-Y-F-IL-M-V-C-DE-K-G-P-NQS-T-A-H-R
17	W-Y-F-I-L-M-V-C-DE-K-G-P-NQS-T-A-H-R
18	W-Y-F-I-L-M-V-C-DE-K-G-P-N-QS-T-A-H-R
19	W-Y-F-I-L-M-V-C-D-E-K-G-P-N-QS-T-A-H-R

**Table 2:** Performance comparison with the state-of-the-art predictor on the benchmark dataset.

Methods	Sn (%)	Sp (%)	Acc (%)	Feature number
Feng et al.	72.04	66.05	66.88	44
Bayes net	38.68	93.55	85.09	90
Random forest	28.09	93.12	80.34	—
AodPred	75.09	74.48	74.79	158
ANPrAod	92.92	98.33	87.53	93

## Data Availability

To facilitate the comparison of our model with previous work, we used the same benchmark dataset collected in the study of Feng et al. (doi:10.1007/s12539-015-0124-9).

## References

[1] Liguori I., Russo G., Curcio F. (2018). Oxidative stress, aging, and diseases. *Clinical Interventions in Aging*.

[2] Pisoschi A. M., Pop A. (2015). The role of antioxidants in the chemistry of oxidative stress: a review. *European Journal of Medicinal Chemistry*.

[3] Shao L., Gao H., Liu Z., Feng J., Tang L., Lin H. (2018). Identification of antioxidant proteins with deep learning from sequence information. *Frontiers in Pharmacology*.

[4] Sun Q., Kong W., Mou X., Wang S. (2019). Transcriptional regulation analysis of Alzheimer's disease based on FastNCA algorithm. *Current Bioinformatics*.

[5] Ao C., Zhou W., Gao L., Dong B., Yu L. (2020). Prediction of antioxidant proteins using hybrid feature representation method and random forest. *Genomics*.

[6] Zhai Y., Chen Y., Teng Z., Zhao Y. (2020). Identifying antioxidant proteins by using amino acid composition and protein-protein interactions. *Frontiers in Cell and Development Biology*.

[7] Meng C., Jin S., Wang L., Guo F., Zou Q. (2019). AOPs-SVM: a sequence-based classifier of antioxidant proteins using a support vector machine. *Frontiers in Bioengineering and Biotechnology*.

[8] Zuo Y., Chang Y., Huang S., Zheng L., Yang L., Cao G. (2019). iDEF-PseRAAC: identifying the defensin peptide by using reduced amino acid composition descriptor. *Evolutionary Bioinformatics*.

[9] Feng P., Chen W., Lin H. (2016). Identifying antioxidant proteins by using optimal dipeptide compositions. *Interdisciplinary Sciences*.

[10] Fu X., Cai L., Zeng X., Zou Q. (2020). StackCPPred: a stacking and pairwise energy content-based prediction of cell-penetrating peptides and their uptake efficiency. *Bioinformatics*.

[11] Tan J. X., Li S. H., Zhang Z. M. (2019). Identification of hormone binding proteins based on machine learning methods. *Mathematical Biosciences and Engineering*.

[12] Han P., Zhang X., Norton R. S., Feng Z.-P. (2006). Predicting disordered regions in proteins based on decision trees of reduced amino acid composition. *Journal of Computational Biology*.

[13] Liu B., Xu J., Lan X. (2014). iDNA-Prot|dis: identifying DNA-binding proteins by incorporating amino acid distance-pairs and reduced alphabet profile into the general pseudo amino acid composition. *PLoS One*.

[14] Feng P., Ding H., Lin H., Chen W. (2017). AOD: the antioxidant protein database. *Scientific Reports*.

[15] Liang Z. Y., Lai H. Y., Yang H. (2017). Pro54DB: a database for experimentally verified sigma-54 promoters. *Bioinformatics*.

[16] Zhang T., Tan P., Wang L. (2017). RNALocate: a resource for RNA subcellular localizations. *Nucleic Acids Research*.

[17] Raghunath A., Nagarajan R., Perumal E. (2020). ZFARED: a database of the antioxidant response elements in zebrafish. *Current Bioinformatics*.

[18] Zuo Y., Lv Y., Wei Z., Yang L., Li G., Fan G. (2015). iDPF-PseRAAAC: a web-server for identifying the defensin peptide family and subfamily using pseudo reduced amino acid alphabet composition. *Plos One*.

[19] Chang C. C., Lin C. J. (2011). LIBSVM. *ACM Transactions on Intelligent Systems and Technology*.

[20] Dao F. Y., Lv H., Zhang D., Zhang Z. M., Liu L., Lin H. (2020). DeepYY1: a deep learning approach to identify YY1-mediated chromatin loops. *Briefings in Bioinformatics*.

[21] Dao F. Y., Lv H., Zulfiqar H. (2020). A computational platform to identify origins of replication sites in eukaryotes. *Briefings in Bioinformatics*.

[22] Zhang D., Xu Z. C., Su W. (2020). iCarPS: a computational tool for identifying protein carbonylation sites by novel encoded features. *Bioinformatics*.

[23] Zuo Y., Li Y., Chen Y., Li G., Yan Z., Yang L. (2017). PseKRAAC: a flexible web server for generating pseudo K-tuple reduced amino acids composition. *Bioinformatics*.

[24] Yan J., Bhadra P., Li A. (2020). Deep-AmPEP30: improve short antimicrobial peptides prediction with deep learning. *Molecular Therapy - Nucleic Acids*.

[25] Zheng L., Huang S., Mu N. (2019). RAACBook: a web server of reduced amino acid alphabet for sequence-dependent inference by using Chou's five-step rule. *Database*.

[26] Zheng L., Liu D., Yang W., Yang L., Zuo Y. (2020). RaacLogo: a new sequence logo generator by using reduced amino acid clusters. *Briefings in Bioinformatics*.

[27] ValizadehAslani T., Zhao Z., Sokhansanj B. A., Rosen G. L. (2020). Amino acid k-mer feature extraction for quantitative antimicrobial resistance (AMR) prediction by machine learning and model interpretation for biological insights. *Biology*.

[28] He S., Guo F., Zou Q., HuiDing (2021). MRMD2.0: a Python tool for machine learning with feature ranking and reduction. *Current Bioinformatics*.

[29] Patil K., Chouhan U. (2019). Relevance of machine learning techniques and various protein features in protein fold classification: a review. *Current Bioinformatics*.

[30] Zou Q., Wan S., Ju Y., Tang J., Zeng X. (2016). Pretata: predicting TATA binding proteins with novel features and dimensionality reduction strategy. *BMC Systems Biology*.

[31] Lin H., Ding H. (2011). Predicting ion channels and their types by the dipeptide mode of pseudo amino acid composition. *Journal of Theoretical Biology*.

[32] Tang H., Zhao Y. W., Zou P. (2018). HBPred: a tool to identify growth hormone-binding proteins. *International Journal of Biological Sciences*.

[33] Feng C. Q., Zhang Z. Y., Zhu X. J. (2019). iTerm-PseKNC: a sequence-based tool for predicting bacterial transcriptional terminators. *Bioinformatics*.

[34] Bradley A. P. (1997). The use of the area under the ROC curve in the evaluation of machine learning algorithms. *Pattern Recognition*.

[35] Jiao Y., Du P. (2016). Performance measures in evaluating machine learning based bioinformatics predictors for classifications. *Quantitative Biology*.

[36] Zhang D., Chen H.-D., Zulfiqar H. (2021). iBLP: an XGBoost-based predictor for identifying bioluminescent proteins. *Computational and Mathematical Methods in Medicine*.

[37] Zhang Z.-Y., Yang Y.-H., Ding H., Wang D., Chen W., Lin H. (2021). Design powerful predictor for mRNA subcellular location prediction in Homo sapiens. *Briefings in Bioinformatics*.

[38] Dao F. Y., Lv H., Wang F. (2019). Identify origin of replication in Saccharomyces cerevisiae using two-step feature selection technique. *Bioinformatics*.

[39] Solis A. D. (2015). Amino acid alphabet reduction preserves fold information contained in contact interactions in proteins. *Proteins*.

[40] Hsu C.-W., Lin C.-J. (2002). A comparison of methods for multiclass support vector machines. *IEEE Transactions on Neural Networks*.

[41] Campbell C. (2002). Kernel methods: a survey of current techniques. *Neurocomputing*.

[42] Zhang J., Liu B. (2019). A review on the recent developments of sequence-based protein feature extraction methods. *Current Bioinformatics*.

